RETRACTED

# Mechanism of Sevoflurane Anesthesia under Hypothermic Cardiopulmonary Bypass on Postoperative Atrial Fibrillation Rhythm in Patients Undergoing Mitral Valve Replacement

**DOI:** 10.1155/2022/5312897

**Published:** 2022-06-28

**Authors:** Hao Che, Yufang Lv, Fang Yao, Fang Zhao, Liyun Zhao

**Affiliations:** ^1^Department of Anesthesiology, Beijing Anzhen Hospital of Capital Medical University, Beijing 100029, China; ^2^Department of Anesthesiology, Chaoyang City Second Hospital, Chaoyang, 122000 Liaoning Province, China

## Abstract

**Objective:**

It was to investigate the mechanism of atrial fibrillation after mitral valve replacement under extracorporeal circulation in patients with rheumatic heart disease under sevoflurane anesthesia maintenance and to provide scientific and effective basis for clinical treatment.

**Methods:**

Forty patients with rheumatic heart disease who underwent mitral valve replacement were randomly rolled into group I (sinus rhythm of propofol anesthesia, *n* = 10), group II (atrial fibrillation rhythm of propofol anesthesia, *n* = 10), group III (sinus rhythm of sevoflurane anesthesia, *n* = 10), and group IV (atrial fibrillation rhythm of sevoflurane anesthesia, *n* = 10). Inflammatory factors, free tissue of right atrium, and incidence of postoperative atrial fibrillation were compared among all groups.

**Results:**

(i) The serum levels of NT-proBNP, CRP, sST-2, IL-6, TNF-*α*, and TGF-*β*1 in group II were higher than those in group I, group III, and group IV, and the indexes in group III were higher than those in group IV (*P* < 0.05). (ii) The relative expression levels of PLB, CaMK II, Bax, and TP53 in the free tissue of right atrium in group II were higher than those in group I, III, and IV, and the index levels in group IV were higher than those in group III (*P* < 0.05). (iii) The incidence of postoperative atrial fibrillation in group III (0.00%) was significantly lower than that in group I (30%), group II (50%), and group IV (40.0%), and group II (50%) was the highest (*P* < 0.05).

**Conclusion:**

The maintenance of sevoflurane anesthesia can improve the inflammatory response and myocardial tissue autophagy in patients with sinus rhythm and atrial fibrillation rhythm and can reduce the incidence of postoperative atrial fibrillation in patients.

## 1. Introduction

Atrial fibrillation is the most common arrhythmia in clinical practice, and its incidence tends to increase with age [1]. The incidence of atrial fibrillation is high in patients with rheumatic heart disease, and when severe, it can evidently affect the quality of life of patients [2]. At present, the only radical treatment for rheumatic heart disease is mitral valve replacement, which has good clinical application effect [3]. However, mitral valve replacement has high surgical risk, slow prognosis, and heart failure. When the optimal surgical opportunity is missed, patients' atrial fibrillation and left atrial enlargement are difficult to be effectively alleviated [4]. In addition, during the onset of atrial fibrillation, patients are prone to thrombosis in the atria, which leads to severe and concurrent occurrence of cerebral embolism and systemic circulation embolism, thus, having a high disability rate and fatality rate [5]. Therefore, it is very important to alleviate the onset of atrial fibrillation in patients. Atrial fibrillation is maintained by drug therapy to maintain sinus rhythm, and the probability of embolization after atrial fibrillation is reduced by ablative therapy, anticoagulation therapy, and other methods [6]. In recent years, studies suggested that electrical remodeling of the atria can lead to shortening, prolonging, or incongruity of the effective refractory period. Remodeling can trigger the delay of electrical signal conduction in the atria and then cause the dysfunction of atrial contraction function [7, 8]. In addition, myocardial fibrosis also plays an important role in atrial remodeling [9]. The main forms of myocardial fibrosis are the deposition of fibrous tissue in the interstitium of cardiomyocytes and replacement/repair fibrosis after apoptosis of cardiomyocytes. In summary, atrial remodeling plays an important role in the occurrence of atrial fibrillation.

RETRACTED

Recent studies confirmed that inflammatory response is also associated with the occurrence and maintenance of atrial fibrillation [10, 11]. In surgery, sevoflurane inhalation anesthesia can effectively reduce the incidence of atrial fibrillation and other rapid heart rate disorders in patients during or after surgery, so it has a certain effect of drug defibrillation [12]. Sevoflurane does not stimulate the respiratory tract and does not increase airway secretions, but can easily cause respiratory depression and reduce the levels of insulin and glucagon [13]. Propofol, a short-acting intravenous anesthetic, is administered intravenously to put patients to sleep quickly and smoothly. However, the analgesic effect of this drug is weak and will cause adverse reactions such as respiratory depression, decreased blood pressure, and decreased intracranial pressure [14]. At present, there is a lack of clinical comparison on the application effect of the two anesthetics.

Therefore, this study is aimed at exploring the effects of sevoflurane and propofol anesthesia on the incidence of atrial fibrillation in patients undergoing mitral valve replacement under hypothermia cardiopulmonary bypass and at exploring the changes of sevoflurane on the inflammatory response and myocardial cell apoptosis in patients. The mechanism of action of sevoflurane on myocardial protection of patients undergoing mitral valve replacement under CPB was explored, to provide effective research basis for improving surgical effect and prognosis of patients.

RETRACTED

## 2. Materials and Methods

### 2.1. General Information

Forty patients with rheumatic heart disease who underwent mitral valve replacement in X Hospital from June 2017 to June 2020 were selected as the study subjects. Patients were randomly rolled into group I (sinus rhythm group under propofol anesthesia (*n* = 10)), group II (atrial fibrillation group under propofol anesthesia (*n* = 10)), group III (sinus rhythm group under sevoflurane anesthesia (*n* = 10)), and group IV (atrial fibrillation group under sevoflurane anesthesia (*n* = 10)) according to random number table method. General data, cardiac function grades, valve regurgitation before and after surgery, cardiac function indicators, and the incidence of atrial fibrillation one day after surgery were collected. Inclusion criteria: (i) patients diagnosed with chronic rheumatic heart disease and mitral stenosis by clinical signs, medical history, and imaging examination; (ii) patients with a history of atrial fibrillation heart rhythm at least six months; (iii) there was no severe mitral regurgitation. Exclusion criteria: (i) patients with complicated infective endocarditis; (ii) patients with diabetes, hypertension, coronary heart disease, or severe organ insufficiency; (iii) patients with preoperative treatment history of calcium channel blockers; (iv) patients with aortic stenosis; (v) patients with mitral valve severe regurgitation; (vi) women with active liver disease, pregnancy, or lactation; (vii) patients with malignant tumors or immune system diseases.

This study had been reviewed and approved by the medical ethics committee, and all patients included in the study had been aware of the trial process and signed the informed consent.

### 2.2. Treatment Methods

All patients underwent surgical treatment under general anesthesia and hypothermia external circulation. In addition, the surgical incision was located at the midline of the sternum, and cardiopulmonary bypass was established. Routine monitoring of pulse oxygen saturation and noninvasive blood pressure was required from the time the patient entered the operating room. Invasive blood pressure monitoring was implemented via radial artery puncture and a five-lead electrocardiogram. After endotracheal intubation, end-tidal carbon dioxide partial pressure and nasopharyngeal temperature were monitored. The central venous pressure was monitored by internal jugular vein puncture and catheterization. All patients received 0.1 mg/kg midazolam + 0.3 mg/kg etomidate + 0.005 mg/kg fentanyl + 0.15 mg/kg vecuronium for induction of anesthesia. Patients in groups I and II were then given 2% propofol to maintain anesthesia. Patients in groups III and IV received 2% sevoflurane for maintenance anesthesia. All patients in each group needed intermittent infusion of fentanyl and vecuronium during maintenance anesthesia. The bispectral index (BIS) was used to detect the depth of anesthesia, and the BIS was maintained at about 40 ± 5.

RETRACTED

After an incision was made in the middle of the sternum, the pericardium was opened, and 300 IU/kg heparin was administered. Catheterization of the aorta and vena cava and cardiopulmonary bypass was performed after the coagulation time of the whole blood exceeded 480 s. The central venous pressure was required to be maintained during surgery. If the patient appeared hypotension, it was necessary to timely supplement deoxyadrenalin for pressor treatment. After surgery, twelve-lead electrocardiogram was used to diagnose atrial fibrillation rhythm.

### 2.3. Detection of Serum Biochemical Indexes

Fasting cubital vein blood was collected and placed in a refrigerator at -20°C for 60 min after anticoagulation treatment, followed by centrifugation at 3,000 rpm for 10 min, and supernatant was taken. The electrochemiluminescence double antibody sandwich immunoassay was adopted to determine the level of serum midbrain natriuretic peptide N-terminal precursor hormone (NT-probNP), and the kit was purchased from Roche. Enzyme-linked immunosorbent assay (ELISA) (Thermo, USA, MultiskanFC microplate analyzer) was used to detect C-reactive protein (CRP), somatostatin subtype receptor 2 (SST-2), interleukin (IL) -6, tumor necrosis factor (TNF-*α*), and transforming growth factor (TGF-*β*1) in serum of patients, following the instructions.

### 2.4. Real-Time Quantitative PCR Detection

When mitral valve replacement was performed and cardiopulmonary bypass was established, a small amount of free wall tissue of the right atrium was taken, rinsed with phosphoric acid buffer, and stored in liquid nitrogen. After grinding of the tissues, an appropriate amount of Trizol reagent was added to extract total RNA, and the concentration, purity, and integrity were detected. Reverse transcription of cDNA was performed according to the instructions of the cDNA reverse transcription kit (Takara, Japan). Phospholamban (PLB), calmodulin-dependent protein kinase II (CaMK-II), Bax, and tumor protein 53 (TP53) quantitative detection primers were designed and synthesized, as shown in Table 1. The target gene expression was detected according to the instructions of the TB Green® Premix Ex Taq™ test kit (Takara, Japan). The PCR products were detected by 2% agarose gel electrophoresis imaging. 2% agarose gel with a thickness of 3 mm was taken, 5-10 *μ*L PCR reaction solution containing 3 *μ*L bromophenollan solution was added, medium voltage electrophoresis apparatus was applied, and 0.5 × TBE working solution was given under the power supply. Then, the electrophoresis lasted for 50 min under the voltage of 80 V. The test was carried out on the quartz glass table of the UV transmittance instrument. Using GAPDH gene as internal reference, 2-^△△Ct^ was used to detect the relative expression level of target gene.

RETRACTED

### 2.5. Statistical Treatment

SPSS 19.0 was employed to arrange the experimental data. The dichotomous variables were represented by frequency (%), and the continuous variables were represented by means ± SD, whose differences were compared by chi-square test and one-way ANOVA, respectively. When *P* < 0.05, there was a significant difference between the two groups.

## 3. Results

### 3.1. Comparison of General Information

Before surgery, the differences among the general information of the four groups of patients were compared in Table 2. It was found that the average age, sex ratio, TC, Cr, UA, LADd, RADd, LVDd, RVDd, LVEF, and cardiac function classification of the patients in each group had no significant difference (*P* > 0.05).

### 3.2. The Effect of Sevoflurane on the Level of Serum Biochemical Indexes in Patients

The differences in serum levels of NT-proBNP, CRP, sST-2, IL-6, TNF-*α*, and TGF-*β*1 in each group of patients were compared before operation (0 h), 3 h after operation, 12 h after operation, and 24 h after operation. The results were shown in Figure 1. With the prolongation of the operation, the serum levels of NT-proBNP, CRP, sST-2, IL-6, TNF-*α*, and TGF-*β*1 in each group reached the highest at 12 h after surgery, and they were all reduced at 24 h after surgery. The differences in serum biochemical index levels of patients in each group at each time point were compared. With 24 hours after operation as an example, compared with group I, the levels of serum indexes of patients in group II were dramatically increased (*P* < 0.05), and the levels of serum indexes of patients in groups III and IV were greatly decreased (*P* < 0.05). Compared with group II, serum levels of patients in group III and group IV were obviously lower (*P* < 0.05). The serum levels of patients in group IV were notably superior to those of group III (*P* < 0.05).

RETRACTED

### 3.3. The Effect of Sevoflurane on the Expression of PLB, CaMK II, Bax, and TP53 in Patients

Real-time fluorescence quantitative PCR was used to detect the relative expression levels of PLB, CaMK II, Bax, and TP53 in the right atrium free tissues of each group of patients. The detection bands were shown in Figure 2. The expression levels of PLB, CaMK II, Bax, and TP53 in the tissues of group II were the highest, while the expression levels of PLB, CaMK II, Bax, and TP53 were the lowest in the tissues of group III.

Subsequently, GAPDH was used as an internal reference gene to calculate the relative expression levels of PLB, CaMK II, Bax, and TP53, and the results were shown in Figure 3. Compared with group I, the expression levels of PLB, CaMK II, Bax, and TP53 in the tissues of group II patients were dramatically increased (*P* < 0.05). The expression levels of PLB, CaMK II, Bax, and TP53 in the tissues of patients in groups III and IV were substantially reduced (*P* < 0.05). In addition, the expression levels of PLB, CaMK II, Bax, and TP53 in the tissues of patients in groups III and IV were obviously lower than those in group II (*P* < 0.05). The expression levels of PLB, CaMK II, Bax, and TP53 in the tissues of the group IV were notably superior to those in the group III (*P* < 0.05).

### 3.4. Comparison of Incidence of Atrial Fibrillation

The difference between the probability of atrial fibrillation in each group of patients was compared during the operation to 24 hours after the end of the operation, and the results were shown in Figure 4. The probability of atrial fibrillation in group I, group II, group III, and group IV was 30.0%, 50.0%, 0.0%, and 40.0%, respectively. Compared with group I (*P* < 0.05), the incidence of atrial fibrillation in group II was dramatically increased, but the incidence of atrial fibrillation in group III was substantially reduced (*P* < 0.05). In addition, the incidence of atrial fibrillation in group III was also substantially reduced compared with group II and group IV (*P* < 0.05).

## 4. Discussion

Atrial fibrillation affects about 2% of the general population, and there are many factors to induce atrial fibrillation [15]. Studies revealed that for every additional ten years of age, the risk of atrial fibrillation increases two times. The incidence of atrial fibrillation in males is 1.5 times higher than that in females [16]. At present, a number of studies concluded that there are many factors triggering atrial fibrillation, mainly including inflammatory response, oxidative stress, and autonomic nervous system imbalance [7, 17]. The underlying mechanism of atrial fibrillation may be related to the abnormality of focal potential and arrhythmia, but the specific mechanism remains unclear and uncertain. Studies confirmed that sevoflurane inhalation anesthesia can effectively reduce the incidence of atrial fibrillation in patients, with certain drug defibrillation effect [18]. Therefore, the effects of sevoflurane and propofol anesthesia maintenance on serum NT-proBNP, CRP, sST-2, IL-6, TNF-*α*, and TGF-*β*1 levels in patients undergoing mitral valve replacement surgery were analyzed. NT-proBNP is a type of peptide hormone. When atrial pressure tension increases, the level of NT-proBNP will also increase [19]. IL-6 is mainly produced by T cells and macrophages, which can induce the expression of inflammatory response proteins in the acute phase, such as TNF-*α*. CRP, TNF-*α*, and TGF-*β*1 all belong to a class of inflammatory mediators [20]. Studies pointed out that there will be more obvious inflammation in the myocardial tissue of patients with atrial fibrillation [21]. SST-2 belongs to the family of interleukins, which can help the immune response of T cells after binding to IL-33 and inhibit the fibrosis and apoptosis of myocardial tissue [22]. The results showed that compared with patients with sinus rhythm, postoperative serum NT-proBNP, CRP, sST-2, IL-6, TNF-*α*, and TGF-*β*1 levels in patients with atrial fibrillation all increased to varying degrees, which confirmed the relationship between the occurrence of atrial fibrillation and the body's inflammatory response, indicating that the inflammatory response can promote the occurrence of postoperative atrial fibrillation in patients [23]. Compared with the maintenance of propofol anesthesia, sevoflurane used for maintenance of anesthesia in patients with atrial fibrillation substantially reduced serum NT-proBNP, CRP, sST-2, IL-6, TNF-*α*, and TGF-*β*1 levels after maintenance. Sevoflurane is a kind of volatile anesthetic, and its effect on myocardial protection is evidently better than that of intravenous anesthetics [24]. The results confirmed that sevoflurane anesthesia can greatly reduce the postoperative inflammatory response in patients.

RETRACTED

Real-time fluorescence quantitative PCR technology was used to detect the changes in the expression levels of PLB, CaMK II, Bax, and TP53 mRNA in the free tissues of the patient's right atrium. In myocardial tissue, PLB can inhibit the activity of the sarcoplasmic reticulum calcium pump, thereby inhibiting the entry of calcium ions into the sarcoplasmic reticulum [25]. CaMK II phosphorylation can form pentamers with PLB, and the two factors can mutually regulate the release of calcium ions during myocardial diastole and systole and then participate in the occurrence of arrhythmia such as atrial fibrillation [26]. Moreover, there is also a close relationship between atrial fibrillation and the apoptosis of cardiomyocytes. Bax is an important factor regulating cell apoptosis, which can promote cell apoptosis [27]. TP53 can cause cell apoptosis and cardiac dysfunction [28]. It was found that compared with patients with sinus rhythm, the expression levels of PLB, CaMK II, Bax, and TP53 mRNA in the free tissues of the right atrium in patients with atrial fibrillation were dramatically increased after surgery. It was revealed that there were phenomena such as increased release of calcium ions from cardiomyocytes and cardiomyocyte apoptosis in patients with atrial fibrillation [29]. Compared with the propofol anesthesia group, the expression levels of PLB, CaMK II, Bax, and TP53 mRNA in the atrial free tissues of patients with atrial fibrillation after sevoflurane anesthesia were substantially reduced. It was also found that after sevoflurane anesthesia, the probability of atrial fibrillation recurrence in patients with atrial fibrillation was 0.0%. Therefore, sevoflurane anesthesia can evidently improve postoperative atrial fibrillation and inflammation in patients undergoing mitral valve replacement under hypothermic cardiopulmonary bypass, and the effect was better than propofol anesthesia.

## 5. Conclusion

The effects of sevoflurane and propofol anesthesia on atrial fibrillation in patients undergoing mitral valve replacement were investigated. The results showed that sevoflurane anesthesia could significantly reduce the postoperative inflammatory response, the release of calcium ions, and apoptosis of cardiomyocytes in patients with atrial fibrillation, and significantly reduce the incidence of postoperative atrial fibrillation. However, only clinical data were used to analyze the mechanism of sevoflurane in patients with atrial fibrillation after mitral valve replacement. The underlying regulatory mechanism is still unclear; therefore, the relationship between sevoflurane and postoperative atrial fibrillation will be further explored through animal or cell studies. However, through this study, it is concluded that sevoflurane has a good development prospect in clinical surgical anesthesia for patients with atrial fibrillation, and it is worthy of further study.

## Figures and Tables

**Figure 1:** Comparison of differences in serum biochemical index levels of patients in each group. Note: (a) NT-proBNP level; (b) CRP level; (c) sST-2 level; (d) IL-6 level; (e) TNF-*α* level; (f) TGF-*β*1 level. Compared to group I, ^∗^*P* < 0.05; compared with group II, ^#^*P* < 0.05; compared with group III, ^&^*P* < 0.05.

RETRACTED

**Figure 2:** PCR diagram of the detection of the expression level of each target gene.

**Figure 3:** Statistics of the relative expression level of each target gene. Note: (a) the relative expression level of PLB; (b) the relative expression level of CaMK II; (c) the relative expression level of Bax; (d) the relative expression level of TP53. Compared to group I, ^∗^*P* < 0.05; compared with group II, ^#^*P* < 0.05; compared with group III, ^&^*P* < 0.05.

**Figure 4:** Statistics of the incidence of atrial fibrillation in each group of patients. (“∗” meant that compared with group III, the incidence of atrial fibrillation in group I, II, and IV was higher, and there was a statistical difference (*P* < 0.05).)

**Table 1:** Quantitative primers of target genes.

Gene	Primer (5′ →3′)	Product (bp)
PLB	F: AGAGTGGATGCAGGAAGAGAT	235
	R: AGAGCCCAGAGAAGGTTTGAT	

CaMK II	F: ACTGGCGTCACGTTGTACTG	127
	R: CCTCGCTGATTTCTGGCTCC	

Bax	F: CCCGAGAGGTCTTTTTCCGAG	155
	R: CCAGCCCATGATGGTTCTGAT	

TP53	F: ACTTGTCGCTCTTGAAGCTAC	113
	R: GATGCGGAGAATCTTTGGAACA	

GAPDH	F: TGTGGGCATCAATGGATTTGG	116
	R: ACACCATGTATTCCGGGTCAAT	

**Table 2:** Comparison of general information of patients in each group.

Item	Group I (*n* = 10)	Group II (*n* = 10)	Group III (*n* = 10)	Group IV (*n* = 10)
Age (years old)	60.17 ± 5.33	61.20 ± 6.18	62.07 ± 5.74	61.58 ± 4.39
Male (*n*/%)	4/40.0	5/50.0	5/50.0	5/50.0
TC (mmol/L)	4.77 ± 0.43	4.78 ± 0.41	4.77 ± 0.50	4.80 ± 0.49
Cr (mg/dL)	85.09 ± 0.67	85.36 ± 1.88	86.05 ± 1.52	86.11 ± 2.13
UA (mg/dL)	323.25 ± 91.25	330.62 ± 97.14	331.29 ± 89.13	328.43 ± 86.47
LADd (mm)	46.31 ± 5.28	50.33 ± 8.97	47.05 ± 9.03	50.84 ± 10.26
RADd (mm)	36.07 ± 5.15	40.12 ± 6.36	37.11 ± 6.17	40.97 ± 6.05
LVDd (mm)	51.36 ± 8.02	52.11 ± 8.93	51.02 ± 7.11	52.03 ± 8.21
RVDd (mm)	36.85 ± 6.07	38.54 ± 6.17	36.90 ± 5.22	38.46 ± 6.28
LVEF (%)	64.72 ± 8.36	60.14 ± 11.07	62.08 ± 8.14	59.08 ± 10.36
Heart function (*n*/%)				
Grade I	1/10.0	0/0.0	1/10.0	0/0.0
Grade II	4/40.0	4/40.0	3/30.0	4/40.0
Grade III	5/50.0	6/60.0	6/60.0	5/50.0
Grade IV	0/0.0	0/0.0	0/0.0	0/0.0

TC: total cholesterol; Cr: creatinine; UA: uric acid; LADd: left atrial end-diastolic diameter; RADd: right atrial end-diastolic diameter; LVDd: left ventricular end-diastolic diameter; RVDd: right ventricular end-diastolic diameter; LVEF: left ventricular ejection fraction.

## Data Availability

The data used to support the findings of this study are included within the article.
